RETRACTED

# Generalized Zero-Adjusted Models to Predict Medical Expenditures

**DOI:** 10.1155/2021/5874275

**Published:** 2021-12-13

**Authors:** Xin Xu, Tao Ye, Dongxiao Chu

**Affiliations:** ^1^School of Finance, Capital University of Economics and Business, Beijing 100070, China; ^2^School of Banking and Finance, University of International Business and Economics, Beijing 100029, China

## Abstract

In healthcare research, medical expenditure data for the elderly are typically semicontinuous and right-skewed, which involve a point mass at zero and may exhibit heteroscedasticity. The problem of a substantial proportion of zero values prevents traditional regression techniques based on the Gaussian, gamma, or inverse Gaussian distribution, which may lead to understanding the standard errors of the parameters and overestimating their significance. A common way to counter the problem is using zero-adjusted models. However, due to the right-skewness in the nonzeros' response, conventional zero-adjusted models such as zero-adjusted gamma, zero-adjusted Inverse Gaussian, and classic Tobit may not perform well. Here, we firstly generalize those three types of the conventional zero-adjusted model to solve the problem of right-skewness in health care. The generalized zero-adjusted models are very flexible and include the zero-adjusted Weibull, zero-adjusted gamma, zero-adjusted inverse Gaussian, and classic Tobit models as their special cases. Using the Chinese Longitudinal Healthy Longevity Survey, we find that, according to the AIC, SBC, and deviance criteria, the zero-adjusted generalized gamma model is the best one of these generalized models to predict the odds of zero cost accurately. In order to depict the predictors affecting the amount expenditure, we further discuss the situations where the mean, dispersion of a nonzero amount expenditure and model the probability of a zero amount of ZAGG in terms of predictor variables using suitable link functions, respectively. Our analysis shows that age, health, chronic diseases, household income, and residence are the main factors influencing the medical expenditure for the elderly, but the insurance is not significant. To the best of our knowledge, little study focused on these situations, and this is the first time.

## 1. Introduction

The ageing of the population is a universal law of the development of human society. According to the definition of the United Nations, if more than 10% of the total population of a country or region is seniors over 60 or over 7% are seniors over 65. The country or region has entered an ageing society. At present, most countries in the world, including the United States, the United Kingdom, and Japan, are about to experience the effects of population ageing. China has no exception and is also facing the complex ageing situation. The proportion of the population over 60 in China has increased from 10% in 1999 to 18% in 2019, nearly doubling in the next twenty years. The weakening of the physiological functions of the elderly will naturally increase their chances of illness, leading to an increase in the demand for health services, which in turn brings about a large number of health and medical security problems for the elderly. Statistics from the China Health Commission showed that approximately 17% of the elderly consume nearly 70% of medical expenses. In addition, the ageing of the population will also inevitably bring about an increase in the life expectancy of the population. Experience has shown that chronic diseases are naturally associated with ageing. Therefore, the ageing population will result in a substantial increase in the prevalence of various chronic diseases. Ingmar et al. [1] discovered exceeding 60% of aged 65 and older had three or more coexisting chronic diseases in Germany. More than 180 million older adults in China suffer from chronic diseases, and the coexistence of multiple diseases is common. According to the statistics of China's health and family planning, the medical expenditure of chronic diseases accounts for more than 70% of the health expenditure. However, due to the imperfections of China's existing medical security system, the out-of-pocket medical expense is relatively large, and medical security is insufficient [2, 3]. When the elderly's out-of-pocket medical expenditure reached or exceeded their ability to pay, some elderly people are not going to see the doctor after they become ill. Compared with other diseases, chronic diseases have the characteristics of insidious onset and long course, which will not only significantly increase the medical expenditure of the elderly [4, 5] but also cause some older adults to fail to receive medical treatment for minor illnesses. Therefore, accurate prediction of medical expenditure for the elderly will not only help the elderly arrange their consumption expenditure reasonably and improve their health status but also be advantageous to the country allocating medical resources more effectively.

RETRACTED

Nevertheless, due to the different personal economic conditions of different elderly groups, they will have differences in medical expenditures after they fall ill. These phenomena will lead to a large number of zero consumption expenditures in the medical expenditure data of the elderly [6, 7], which also will result in right-skewed problems in the distribution of medical consumption data. Because of the point mass at zero and skewness, these problems can hardly be taken into account by traditional regression models such as Poisson, OLS, and gamma models. Ignoring these phenomena would lead to misspecified regression-based estimators and overestimated/underestimated effects. In order to predict more accurately, the medical expenses of the elderly new models need to be proposed. The aim of this paper is to propose a type of generalized zero-adjusted model to better fit the semicontinuous data, explore the influencing factors of elderly's medical expense, use this type of model to predict the amount of medical consumption of the elderly, and compare the results with conventional models.

The specific contributions of this paper include the following: (1) three types of generalized zero-adjusted models such as zero-adjusted generalized gamma model, zero-adjusted generalized inverse Gaussian model, and generalized zero-adjusted Tobit model for predicting the medical expenditure were proposed which included many traditional models and have not been used in health economic cost data modelling before. (2) Selected the best model zero-adjusted generalized gamma model according to different criteria and explored the marginal effects of predictors of medical expenditures. (3) Discovered the relationship between the dispersion of medical expenditure and explanatory variables due to the heterogeneity of variance.

The rest of this paper is organized as follows: detailed literature and related work are given in Section 2. Conventional zero-adjusted models and generalized zero-adjusted models are highlighted in Section 3. Numerous experimental results and comparisons of different models are suggested in Sections 4 and 5. Discussion is shown in Section 6. In the end, conclusions are summarized, and future research is presented in Section 7.

## 2. Related Works

There was much literature about modelling health care costs, although the health economist or health services researcher faced several difficulties. One type of published approaches for the medical expenditure involved modelling the cost using ordinary squares regression directly [8, 9]. Although the ordinary least squares model was used, this method was criticized because the distribution of strictly positive health expenditures was typically skewed, kurtotic (thick-tailed), and heteroskedastic, exhibiting a nonconstant variance that increased with expenditures [10]. These properties make the traditional approach, such as ordinary least squares(OLS) estimation biased and inefficient. Therefore, lots of work had been done on the problems of modelling medical expenditure. In order to solve the right-skewed of the medical expenditure data, Jones transformed the dependent variable using a log transformation to reduce the effect of extreme observations and right skewness and improved the goodness of fit [11]. Manning and Mullahy assumed the medical expenditures to be distributed to an exponential function of the explanatory variables and used log ordinary least squares and the gamma model with a log link to find a more robust alternative estimator than the OLS regression [12]. However, such transformations were likely to be problematic in heteroskedastic errors on the transformed scale [13, 14]. Alternately, there was a large and growing literature on using inherently nonlinear specifications to model medical expenditures, which benefited from estimating effects on the natural scale of costs. The generalized linear model (GLM) and exponential conditional mean models were considered. The generalized linear model was first proposed by Nelder and Wedderburn in the 70s last century and has been widely applied in many fields as once proposed [15]. The generalized linear model assumed that the dependent variable obeyed a type of exponential distribution family, which included many common distributions such as Poisson and normal and supposed the variance of the random error term was not required to be equal. Within the GLM family, it was usual to make assumptions about the functional form of the mean and variance of the distribution. Although the generalized linear model could effectively deal with the problem of heteroscedasticity, it perhaps failed to account explicitly for the issues of skewness and the fat tail, which had implications for the efficiency and robustness of estimators [16]. More flexible distributions for a greater range of estimated skewness and kurtosis coefficients were explored. Manning et al. proposed the generalized gamma models (GGM) to solve the problem of healthcare costs. The GGM model included important parametric distributions as nested and special cases, such as the gamma (GA) and log-normal (LN) distribution. Each model had been selected to model healthcare costs in lots of literature [14]. Because the GGMs was also a special limiting case of the generalized beta of the second kind (GB2), Jones investigated GB2 as part of a comparison of many different methods for modelling US healthcare costs. Mullahy [16]considered the use of the Singh–Maddala distribution (SM) in order to control the heavy right-hand tail of cost data, which was also nested within the GB2.

RETRACTED

Where the censored approach to medical expenditure was concerned, the Tobit regression using a single distribution had been suggested as one of the methods to be used for modelling [17]. In Tobit regression, there was an assumption about the response variable based on a zero-truncated normal distribution. Obviously, the constant variance was assumed in this linear regression setting, and the response variable was right-skewed, which was inadequate for medical expenditure data. Therefore, the Gaussian assumption might not be suitable for fitting medical expenditure with the Tobit model. The censored Gamma regression was introduced to overcome the skewed nature of the response [18]. Unfortunately, the Tobit model could not also handle the excess zeros that was a phenomenon that there were more zeros than from the underlying distribution in the medical expenditure data. From the perspective of the data-generating process, semicontinuous medical expenditure data should be considered as arising from two different stochastic processes. Firstly, the patients might choose whether to see a doctor according to their health status, severity of illness, financial burden, and other reasons, which governed the occurrence of zeros. Secondly, the patients who enjoyed more medical services and higher income were likely to incur higher medical expenditures than those less inclined to use these services, which resulted in extremely asymmetry in the nonzero medical expenditures data. Therefore, a two-part mixture model was an ideal choice for dealing with such data, which separately model the probability of any medical services use and the level of expenditures conditional on use [19]. A large number of papers previously were explicitly devoted to changing the different distributions in the second process, and the binomial distribution or logistic regression model was used frequently in the first process. A log-normal distribution was often chosen to model the positive medical expenditure data [20]. However, many alternative distributions were used to relax the log-symmetry condition imposed by the log-normal distribution because the log-normal distribution was not enough to fit the right-skewed and heavy tail features in the data [21, 22]. To the best of our knowledge, there were many studies about the two-part mixture models used in medical healthcare, but the proposed approach had already been applied in many other fields. Heller et al. used the two-part model to predict the total claim count. The one part was the negative binomial distribution for modelling the claim counts, and the other was the inverse Gaussian for the claim amount that occurred. To estimate the total claim amount [23]. Chai et al. analyzed the semicontinuous arterial calcification scores by introducing a two-part skew log-normal [24, 25]. Liu et al. found that the generalized gamma model provided a superior fit in their analysis of daily alcohol consumption by comparing generalized gamma, log-skew-normal, and box-cox-transformed two-part models [26].

RETRACTED

In recent years, there has been an increase in the use of Tweedie exponential family models to fit semicontinuous data [27]. The Tweedie family of distributions belongs to the exponential family with variance and has a compound Poisson-gamma interpretation with a probability mass at zero. The primary advantage of fitting such Tweedie models was to avoid the two-part model of fitting the frequency and then the amount. It is a single distribution. Frees et al. predicted the insurance claim amount using Tweedie model [28]. Christoph F.K showed the better fit of the Tweedie model by comparing it with two-part models and Tobit model [29]. However, there was also another problem that the proposed Tweedie was not allowed to be fitted explicitly as a function of explanatory variables, according to Smyth and Jorgensen [27].

As an alternative, a recent study has perceived that a zero-adjusted regression model, which mixed discrete and continuous distribution. The discrete distribution of the zero adjusted regression model was represented by the Bernoulli distribution. In contrast, the continuous distribution can be represented by any continuous distribution with a positive range and right skewness. The zero-adjusted model could be regarded as a case of a two-part model. The zero-adjusted model focused more on the probability of zero value. When the probability of the observed zero value was much greater or less than the standard normal distribution, gamma, Weibull, and so on, the zero-adjusted model might be established. These could make the probability of zero occurrences predict more actually. Several applications of zero-adjusted gamma (ZAGA) and zero-adjusted inverse Gaussian (ZAIG) regression models could be found in insurance claims [30, 31]. Nevertheless, it appeared that there had been little work done in health economic cost data modelling before. This study attempted to use zero-adjusted models to predict medical expenditure. Throughout this paper, three types of generalized zero-adjusted models were presented, which comprised the classic Tobit model, ZAGA model and ZAIG model, and could improve the accuracy of the prediction. As far as we knew, there was almost little literature to study on those generalized zero-adjusted models, especially in the field of health care.

## 3. Methodology

### 3.1. Spliced Distribution

This study aims to use models to predict the medical expenditure for the elderly and discover the factors affecting the cost as accurately as possible. One way to dealing with excess zeros and positive skewness is to apply zero-adjusted models. The zero-adjusted model can be considered as a case of spliced distribution. Klugman et al. proposed a splicing method for creating new distributions [32], and it had been applied in modelling heavy tail for operational risk [33]. The density function of an *n-*component spliced distribution is defined as follows [32]:

(1) $$\begin{array}{c} f\left(x\right)=\left\{\begin{array}{c} a_{1}f_{1}\left(x\right),\;\text{if }x\in \;C_{1},\\ a_{2}f_{2}\left(x\right),\;\text{if }x\in \;C_{2},\\ \vdots \\ a_{n}f_{n}\left(x\right),\;\text{if }x\in \;C_{n}. \end{array}\right. \end{array}$$

Here *a*_1_,   ⋯ ,  *a*_*n*_ are positive weights that add up to

(2) $$\begin{array}{c} a_{1}+a_{2}+\cdots +a_{n}=1. \end{array}$$

The functions *f*_*i*_(*x*)(*i*=1,2,…, *n*) are legitimate density functions with all probability on the interval *C*_*i*_: ∫_*C*_*i*__*f*_*i*_(*x*)d*x*=1. The intervals *C*_*i*_ and *C*_*j*_ are mutually exclusive: *C*_*i*_∩*C*_*j*_=Φ, ∀*i* ≠ *j*. The intervals of *C*_*i*_ are also sequentially ordered. That is to say, *x* < *y* if *x* ∈ *C*_*i*_ and *y* ∈ *C*_*j*_ for all *i* < *j*. There is an advantage of the spliced distribution allowing the inclusion of point mass distributions.

RETRACTED

### 3.2. Zero-Adjusted Model

The zero-adjusted model can be regarded as a case of *n*-component spliced distributions when *n* equals 2. The first part has zero expenditure amounts, and the second part has nonzero expenditures, which are assumed to have a continuous distribution that accommodates heavy right-skewed. Let *y*_*i*_ be the expenditures of the *i*th older people, *i*=1,…, *n*. The density function of zero-adjusted distribution may be written as follows:

(3) $$\begin{array}{c} f\left(y|x\right)=\left\{\begin{array}{cc} \pi , & \text{if }y=0,\\ \left(1-\pi \right)\cdot g\left(y|x\right), & \text{if }y>0. \end{array}\right. \end{array}$$

where *g*(*y*) is the density of a continuous, right skewed distribution, and *π* is the probability of zero medical expenditure. The cumulative distribution of a zero-adjusted model (ZAM) can be expressed as

(4) $$\begin{array}{c} F\left(y|x\right)=\pi I_{\left\{y=0\right\}}+\left[\pi +\left(1-\pi \right)G\left(y|x\right)\right]I_{\left\{y>0\right\}}, \end{array}$$

where *I*(·) is an indicator function.

### 3.3. Discrete Part of ZAP

Suppose the probability of an older person is distributed to the Bernoulli. Let *ϖ*_*i*_ be a binary variable indicating the occurrence of the outcome for the older person with medical expenditure in one year and *π*_*i*_ be the probability of the positive medical expenditure, on person *i*. *π*_*i*_ may be a constant such as in equation (3) or be a random variable distributed as follows:

(5) $$\begin{array}{c} f\left(\pi_{i}|x\right)=\pi_{i}^{\varpi_{i}}{\left(1-\pi_{i}\right)}^{1-\varpi_{i}},\;\varpi_{i}=0,1. \end{array}$$

We consider the factors affecting the medical expenditure of the older person and incorporate covariates through the logit link function on *π*_*i*_:

(6) $$\begin{array}{c} \log\frac{\pi_{i}}{1-\pi_{i}}=\eta_{i}. \end{array}$$

The predictor *η*_*i*_ is any form of a function related to factors, but generally is assumed to be a linear system*η*_*i*_=*βX*_*i*_, *β*=(*β*_1_,…, *β*_*p*_), *X*_*i*_ is the vector of factors and *β* is the parameter. According to equation (6), we can predict the probability of medical expenditure for the elderly and determine the influencing factors of their medical decision-making.

RETRACTED

### 3.4. Continuous Part of the Zero-Adjusted Model

Another advantage of spliced distributions is that they allow us to model different parts of a response variable with distributions. There are many candidate distributions for the nonzero heavy-tailed distribution modelling medical expenditures *g*(*y|x*), such as the gamma, inverse Gaussian, log-normal (LN), Weibull (WEI), and log-skew-normal. In this study, we considered two specifications of the spliced distributions. The first specification used the generalized gamma (GG) distribution, which includes the standard gamma, inverse gamma, Weibull, and log-normal distributions as special cases [21, 26]. Another was the generalized inverse Gaussian (GIG) distribution, which includes the inverse Gaussian as a special case and the gamma distribution and inverse gamma distributions as limiting cases [34, 35]. The Tobit distribution was also presented as a baseline comparison for the others, and we generalized the traditional Tobit model.

#### 3.4.1. Gamma Distribution (GA) and Inverse Gaussian Distribution (IG)

There was much work to deal with the problem of skewness and heteroscedasticity by transforming data. The data transformed seemed to be more homogeneous and symmetric. However, homoscedasticity was hardly achieved in fact, which resulted in biased estimation [36, 37]. Instead, we used gamma and inverse Gaussian distribution, which belonged to the generalized models taking into account heteroscedasticity and retaining the original dollar scale of the data. Furthermore, the gamma and inverse Gaussian models could accommodate skewness in the expenditures [38]. The GA model and IG model are included in the generalized linear model, which is mainly composed of three parts:

(1) Systems part: the system part is a linear component which can be seemed like the traditional linear models similarly:
  (7) $$\begin{array}{c} \eta_{i}=x_{i}^{\prime }\beta , \end{array}$$
where *x*_*i*_ is a column vector of covariates for observation *i*, *β* is a column vector of the parameters, and *η*_*i*_ is a column vector of prediction *i*.
(2) Link functions: the link functions *g* is often defined a monotonic and differential, which combines the prediction and the systems part and describes how the expected value of a response *y*_*i*_ is related to the linear predictors:
  (8) $$\begin{array}{c} g\left(\mu_{i}|x\right)=x_{i}^{\prime }\beta , \end{array}$$
where *g* is often defined a log function.
(3) Random parts: the response variables *y*_1_, *y*_2_,…, *y*_*n*_ are independent and distributed from an exponential family which implies there are a relationship between the variance and mean. The general form of exponential family is
  (9) $$\begin{array}{c} f\left(y|\theta ,\varphi \right)=\exp\left[\frac{y\theta -b\left(\theta \right)}{a\left(\varphi \right)}+c\left(y,\varphi \right)\right], \end{array}$$
  where *θ* is called the canonical parameter and represents the location, while *φ* is the dispersion parameter and represents the scale. Many distributions besides GA and IG models belong to the exponential distribution family, for example, normal, Weibull, Poisson, negative binomial distributions, and so on. Because of skewness and heteroscedasticity of the outcome, the densities of the gamma distribution and inverse Gaussian distributions are
  (10) $$\begin{array}{c} \text{gamma}:f\left(y|\mu ,\sigma \right)=\frac{y^{1/\sigma^{2}-1}e^{=y/\left(\sigma^{2}\mu \right)}}{{\left(\sigma^{2}\mu \right)}^{1/\sigma^{2}}\Gamma \left(1/\sigma^{2}\right)},\;y>0,\mu >0,\sigma >0. \end{array}$$

Inverse Gaussian:

(11) $$\begin{array}{c} f\left(y|\mu ,\sigma \right)=\frac{1}{\sqrt{2\pi \sigma^{2}y^{3}}}\exp\left[-\frac{1}{2\mu^{2}\sigma^{2}y}{\left(y-\mu \right)}^{2}\right],\;y,\mu ,\sigma >0. \end{array}$$

Suppose the mean of gamma and inverse Gaussian distribution is *E*(*Y|x*)=*μ*. The variance of gamma distribution is Var(*Y|x*)=*μ*^2^*σ*^2^=(*E*(*Y|x*))^2^*σ*^2^, and *E*(*Y*^*r*^*|x*)=*μ*^*r*^*σ*^2*r*^Γ(1/*σ*^2^+*r*)/Γ(1/*σ*^2^), for *r* > −1/*σ*^2^. The skewness of gamma distribution is 2*σ*, and excess kurtosis is 6*σ*^2^. The gamma distribution is appropriate for positively skewed data. At the same time, the variance of inverse Gaussian distribution is Var(*Y|x*)=*σ*^2^*μ*^3^, and the skewness of inverse Gaussian is 3*μ*^1/2^*σ*, the excess kurtosis is 15*μσ*^2^. The inverse Gaussian distribution is also appropriate for highly positively skewed data. We can see that the variance of response is a function of its mean. Note that the variance function for the inverse Gaussian GLM increases more rapidly with the mean than the gamma GLM.

RETRACTED

#### 3.4.2. Generalized Gamma Distribution (GG)

Although the standard gamma model was fairly robust when we analyzed the positive medical expenditures([39]), it was inefficient when the data were heteroskedastic and heavily right-skewed([14]). The generalized gamma was available among other continuous distributions handling values only on the positive values. The density of the generalized gamma probability distribution is parameterized as a function of *κ*, *μ*, *σ* and is given by [14, 21]

(12) $$\begin{array}{c} f\left(y;k,\mu ,\sigma \right)=\frac{\theta^{\theta }}{\sigma y\sqrt{\theta }\Gamma \left(\theta \right)}\exp\left[z\sqrt{\theta }-\mu \right],\;y\geq 0, \end{array}$$

where *θ*=|*κ*|^−2^*z*=sign(*κ*){ln(*y*) − *μ*}/*σ* and *μ*=*θ*  exp  (|*κ*|*z*)^5^. Because d*z*=(1/*σy*)d*y*, equation (12) could be interpreted as the standard normal distribution (*z*) scale for log-transformed *y*. If *Y* is a random variable distributed to density (12), then its mean was given by

(13) $$\begin{array}{c} E\left(Y|x\right)=\exp\left\{\mu +\frac{\sigma \;\log\left(\kappa^{2}\right)}{\kappa }+\log\left[\Gamma \left(\frac{1}{\kappa^{2}}+\frac{\sigma }{\kappa }\right)\right]-\log\left[\Gamma \left(\frac{1}{\kappa^{2}}\right)\right]\right\}. \end{array}$$

The other moments of the generalized gamma distribution were *m*-th moment = *E*(*Y*^*m*^*|x*)=[exp(*μ*) · *κ*^2*σ*/*κ*^]^*m*^{Γ[(1/*κ*^2^)+(*mσ*/*κ*)]/Γ(1/*κ*^2^)}

And, the variance was

(14) $$\begin{array}{c} \text{variance}=E\left(Y^{2}|x\right)-E^{2}\left(Y|x\right)\\ =\left[\exp\left(\mu \right)\cdot \kappa^{2\sigma /\kappa }\right]\left\{\left[\frac{\Gamma \left(\left(1/\kappa^{2}\right)+\left(2\sigma /\kappa \right)\right)}{\Gamma \left(1/\kappa^{2}\right)}\right]-{\left[\frac{\Gamma \left(\left(1/\kappa^{2}\right)+\left(\sigma /\kappa \right)\right)}{\Gamma \left(1/\kappa^{2}\right)}\right]}^{-2}\right\}. \end{array}$$

The standard gamma, inverse gamma, Weibull, and log-normal distributions were special cases of the generalized gamma distribution. For example, the generalized gamma distribution density reduced to a standard gamma distribution when the shape parameter *θ*=*κ*^−2^ and the scale parameter *ν*=*κ*^2^exp(*μ*),.i.e., the density follows as *f*(*y*; *ν*, *θ*)=(1/*ν*^*θ*^Γ(*θ*))*y*^*θ*−1^exp(−*y*/*ν*), and the mean was exp(*μ*), the variance was *κ*^2^exp(2*μ*). Let *κ*=−*σ*,  *σ* > 0, and the inverse gamma distribution was also obtained. The generalized gamma distribution reduced to an inverse gamma distribution defined as Robert [40], as follows.

*f*(*y*; *ε*, *θ*)=*ε*^*θ*^/Γ(*θ*)(1/*y*)^*θ*+1^exp(−*ε*/*y*), where *ε*=*θ*  exp(*μ*). When the parameter *κ* in equation (12) was fixed at a special value, for example, *κ*=1, density (12) reduces to the probability density function of a Weibull distribution. In addition, if the parameter *κ*⟶0, density (12) reduced to the lognormal distribution, i.e., $f\left(y;\mu ,\sigma \right)=1/\sigma y\sqrt{2\pi }\exp\left\{-{\left(\log\left(y\right)-\mu \right)}^{2}/2\sigma^{2}\right\}$.

RETRACTED

#### 3.4.3. Generalized Inverse Gaussian Distribution (GIG)

We introduced the GIG distribution because the GIG was right-skewed, single-peaked distribution, and had a broader range of shapes. The standard gamma was a case of the GIG. Thus, the GIG could be a more flexible alternative to the standard version of the gamma [39]. The probability density function of the model was parameterized in terms of its mean, dispersion, and shape parameters. The parameterization of the generalized Inverse Gaussian distribution, denoted by GIG(*μ*, *σ*, *ν*), was given by

(15) $$\begin{array}{c} f\left(y;\mu ,\sigma ,\nu \right)={\left(\frac{b}{\mu }\right)}^{\nu }\left[\frac{y^{\nu -1}}{2K_{v}\left(\sigma^{-2}\right)}\right]\exp\left[-\frac{1}{2\sigma^{2}}\left(\frac{by}{\mu }+\frac{\mu }{by}\right)\right], \end{array}$$

for *y* > 0, where *μ* > 0,  *σ* > 0, and −*∞* < *ν* < *∞*. In the above equation (15), *b*=[*K*_*ν*+1_(*σ*^−2^)][*K*_*ν*_(*σ*^−2^)]^−1^ and *K*_*λ*_(*t*) was a modified Bessel function of the second kind [40]: *K*_*λ*_(*t*)=1/2∫_0_^*∞*^*x*^*λ*−1^exp{−1/2*t*(*x*+*x*^−1^)}d*x*. With this parameterization, the mean *E*[*Y|x*]=*μ* and variance Var[*Y|x*]=*μ*^2^[2*σ*^2^/*b*(*ν*+1)+1/*b*^2^ − 1]. The skewness of GIG is

(16) $$\begin{array}{c} \text{skewness}=\mu^{3}\frac{\left[2-6\sigma^{2}/b\left(\nu +1\right)\left(\nu +2\right)\sigma^{4}-2/b^{2}+2\sigma^{2}/b^{3}\left(\nu +2\right)\right]}{{\left[\text{Var}\left(y\right)\right]}^{1.5}},\\ \text{excess kurtosis}=\mu^{4}\frac{\left\{\begin{array}{c} -6+24\sigma^{2}/b\left(\nu +1\right)+4/b^{2}\left[2-\sigma^{4}\left(\nu +1\right)\left(7\nu +11\right)\right]+4\sigma^{2}/b^{3}\left[2\sigma^{4}\left(\nu +1\right)\left(\nu +2\right)\left(\nu +3\right)-4\nu -5\right]+\\ 1/b^{4}\left[4\sigma^{4}\left(\nu +2\right)\left(\nu +3\right)-2\right] \end{array}\right\}}{{\left[\text{Var}\left(y\right)\right]}^{2}}. \end{array}$$

Unlike the majority of models for insurance losses, our general approach could determine the distribution of each risk class based not only on the mean parameter, which was traditionally modelled in terms of covariates but also by using regressors on the dispersion and shape parameters, which described the shape of the GIG distribution. This could be regarded as a very useful property. Additionally, the GIG was a very wide family which included many well-known distributions depending on the estimated values of the dispersion and shape parameters which were modelled as functions of risk factors as was well known. For example, as could be seen, GIG(*μ*, *σ*, −0.5)=IG(*μ*, *σμ*^−1/2^). Therefore, the gamma was a special case of GIG when *b*=1 and *ν*=−1/2. According to Jorgensen [35], *K*_*λ*_(*t*) ~ Γ(*λ*)2^*λ*−1^*t*^−*λ*^ as *t*⟶0, for all *λ* > 0. And, when *σ*⟶*∞*, GIG(*μ*, *σ*, *ν*) had limiting distribution *GA*(*μ*, *ν*^−1/2^) for all *ν* > 0.

RETRACTED

#### 3.4.4. Tobit Distribution

Tobit model was first introduced to model dependent variables with a large fraction of zeros by Tobin [17]. The classic Tobit model assumed that the response was continuous, censored, and normally distributed underlying latent dependent variable *y*^*∗*^. We were interested in designing the latent variable *y*^*∗*^ as a linear regression model:

(17) $$\begin{array}{c} y^{*}=x_{i}^{\prime }\beta +\varepsilon_{i},\;i=1,\ldots ,n\\ y_{i}=\left\{\begin{array}{cc} y^{*}, & \text{if }y^{*}\leq L,\\ L, & \text{if }y^{*}>L, \end{array}\right. \end{array}$$

where *ε* ~ *N*(0, *σ*^2^), *x*_*i*_ is an exogenous and observable explanatory variable. Specifically, if the latent variable*y*^*∗*^ values equal to zero are censored, such as the medical expenditure for the elderly, *L* became zero. Then, the probability of a censored observation sample was

(18) $$\begin{array}{c} \mathrm{Pr}\left(y^{*}\leq L\right)=\mathrm{Pr}\left(x_{i}^{\prime }\beta +\varepsilon \leq L\right)=\Phi \left[\frac{\left(L-x_{i}^{\prime }\beta \right)}{\sigma }\right], \end{array}$$

where Φ(·) was the standard normal cumulative distribution. We could present the truncated expected value of the noncensored observation *y*_*i*_

(19) $$\begin{array}{c} E\left(y_{i}|x_{i},y_{i}>L\right)=x_{i}^{\prime }\beta +\sigma \frac{\phi \left[\left(x_{i}^{\prime }\beta -L\right)/\sigma \right]}{\Phi \left[\left(L-x_{i}^{\prime }\beta \right)/\sigma \right]}, \end{array}$$

where *ϕ*(·) was the density function of standard normal distribution. The classic Tobit model was appropriate when the response had two proprieties: one was that the error *ε* was a normal distribution, and the other was that the negative values of response were censored at *L*.

#### 3.4.5. New Type of Generalized Tobit Distribution

The classic Tobit model was extremely sensitive to its underlying assumptions of normality and homoscedasticity. Therefore, the classic Tobit model should never be fit unless the data were truly normal and censored distribution. However, these were hardly met in real data [41, 42]. Many researchers claimed that a large mass at zero was censored observations when they were not censored, especially for health expenditure data. We provided another generalized Tobit model which was different from the generalized Tobit selection model by Heckman [43]. The Heckman selection model was considered as a generalized Tobit model and mainly connected the two latent outcomes by inverse mills ratio. However, the response variable was assumed to be normally distributed yet. In this paper, we mainly generalized the part where the latent *y*^*∗*^ greater than zero. We selected the *student t* family model in order to compare the classic Tobit model. The *Student t* family model was introduced by Lange et al. [43] and was defined by assuming that *Y*=*μ*+*σT*, where *T* ~ *t*_*v*_ had a standard *t* distribution with *v* degrees of freedom. In this study, the PDF of *Student t* family distribution was given by

(20) $$\begin{array}{c} f_{Y}\left(y;\mu ,\sigma ,v\right)=\frac{1}{\sigma B\left(1/2,\nu /2\right)v^{1/2}}{\left[1+\frac{{\left(y-\mu \right)}^{2}}{\sigma^{2}v}\right]}^{-\left(v+1\right)/2}, \end{array}$$

for −*∞* < *y* < +*∞*, where −*∞* < *μ* < +*∞*, *σ* > 0*ν* > 0, and *B*(*a*, *b*)=Γ(*a*)Γ(*b*)/Γ(*a*+*b*) is the beta function. Note that *T*=(*Y* − *μ*)/*σ* had a standard *t* distribution with *v* degrees of freedom. It was obvious that the *t* distribution had higher kurtosis than the normal distribution and more suitable for modelling leptokurtic data [43]. The excess kurtosis of *t* distribution was 6/*v* − 4(if *v* > 4).

RETRACTED

#### 3.4.6. Modelling the Probability of Zero Expenditures and Expected Nonzero Expenditures in Terms of Explanatory Variables

We focused on the factors influencing the medical decision and the number of medical expenditures but paid attention to the accuracy of prediction. The mean *μ* of regression model determined the number of medical expenditures and the dispersion *σ* could affect the accuracy of prediction. Therefore, we would consider the zero-adjusted regression modes in different cases.

Case 1: when the probability of not seeing a doctor was constant, model (6) degenerated to

(21) $$\begin{array}{c} P\left(y=0|x\right)=\pi , \end{array}$$

(22) $$\begin{array}{c} \log\left(\mu \right)=\eta_{1}=X_{1}^{T}\beta_{1}+\varepsilon , \end{array}$$

where the dispersion *σ* was considered as a constant and not affected by the predictor variables, *X* was the vector of predictors, *β* was the vector of parameters, and *ε* was the error. We used the log link function according to the exponential family [38].

Case 2*:* zero amount was not constant, which was affected by predictor variables, and the dispersion *σ* was still a constant. Then, the probability of a zero medical expenditure and mean is shown as

(23) $$\begin{array}{c} \log\text{ it}\left(\pi \right)=\eta_{2}=X_{2}^{T}\beta_{2}+\varepsilon , \end{array}$$

(24) $$\begin{array}{c} \log\left(\mu \right)=\eta_{3}=X_{3}^{T}\beta_{3}+\varepsilon , \end{array}$$

where *X*, *β*, and *ε* were the same as in equation (21) and (22). Theoretically, the factors that affected the decision-making equation (23) and the amount equation (24) were different. However, many studies assumed that they were the same, that was *X*_2_=*X*_3_.

RETRACTED

Case 3*:* the mean *μ*, dispersion *σ*, and the probability of a zero amount *π* included in zero-adjusted model were all influenced by the predictors, which were modelled in terms of predictor variables using suitable link functions:

(25) $$\begin{array}{c} \log\text{ it}\left(\pi \right)=\eta_{4}=X_{4}^{T}\beta_{4}+\varepsilon , \end{array}$$

(26) $$\begin{array}{c} \log\left(\mu \right)=\eta_{5}=X_{5}^{T}\beta_{5}+\varepsilon , \end{array}$$

(27) $$\begin{array}{c} \log\left(\sigma \right)=\eta_{6}=X_{6}^{T}\beta_{6}+\varepsilon , \end{array}$$

where we could choose the same or different predictors *X* in equations (25)–(27). There had been much literature studying case 1 and case 2, and almost little to discuss case 3 to our best knowledge. In this study, we would analyze the three cases and compare their results.

#### 3.4.7. Maximum Likelihood Estimation

According to the zero-adjusted model, given *n* independent observations *y*_*i*_ for *i*=1,2, ⋯, *n*, the likelihood function was given by

(28) $$\begin{array}{c} L=L\left(\psi |y\right)=\prod_{i=1}^{n}f\left(y_{i}|x\right)=\prod_{i=1}^{n}\left[\sum_{k=1}^{2}\pi_{k}f_{k}\left(y_{i}|x\right)\right], \end{array}$$

where *ψ*=(*θ*, *π*), *y*=(*y*_1_, *y*_2_,…,*y*_*n*_)^*T*^ and *f*_*k*_(*y*_*i*_)=*f*_*k*_(*y*_*i*_*|θ*_*k*_). The log-likelihood function was given by

(29) $$\begin{array}{c} l=l\left(\psi |y\right)=\sum_{i=1}^{n}\log\left[\pi f_{1}\left(y_{i}|x\right)+\left(1-\pi \right)f_{2}\left(y_{i}|x\right)\right]. \end{array}$$

We wished to maximize the log-likelihood *l* concerning *θ* and *π*. Nevertheless, the problem was that the logarithm of the second summation in equation (29) made the solution difficult. In this paper, we used an algorithm provided by Rigby and Stasinopoulos [44] and was based on penalized likelihood estimation.

### 3.5. Model Validation and Verification

#### 3.5.1. Graphic Verification

There were some approaches used for verification and selecting the best model among those models after fitting statistical probability models on the medical expenditures data, which mainly included two types of procedures: the graphical and the numerical approaches [45]. The graphical methods were used to verify whether the model described the systematic part and the independence of the normalized quantile residuals and their normality. In this study, we could obtain the mean, variance, skewness, and kurtosis to check the independence of the normalized quantile residuals and their normality by inspecting the residual versus fitted value plots, residual density plots, and Q-Q plots [44]. To assess the goodness-of-fit of the model, Akaike's information criterion (AIC) [46] and the Schwarz Bayesian criterion (SBC) [47]were considered as the numerical methods for validating and selecting the best model among the verified models. In addition, one goal of this study is to estimate the expected medical cost for individuals (${\overset{\wedge }{y}}_{i}=E\left[y_{i}|x_{i}\right]$). The mean prediction error can be thought as measuring the bias between the predicted outcome and the true response, which is often measured by the mean squared error (MSE).

RETRACTED

#### 3.5.2. Information Criteria

To compare the models and select the best one among the fitted models, we used the AIC, SBC, and the global deviance criteria. The AIC is computed based on the Kullback–Leibler distance in information theory, and the SBC is based on the integrated likelihood of Bayesian theory, which both impose the appropriate penalty on the average of the log-likelihood of models estimated given the number of coefficients estimated. A model with the lowest AIC and SBC values will be selected probably. The AIC is given as follows:

(30) $$\begin{array}{c} \text{AIC}=-2\;\log\left(L\right)+2p, \end{array}$$

where *L* is the likelihood and *p* is the number of parameters in the model. The SBC is defined as:

(31) $$\begin{array}{c} \text{BIC}=-2\;\log\left(L\right)+2p\;\log\left(n\right), \end{array}$$

where *L* and *p* are the same as in AIC and *n* is the sample size. As suggested by Rigby and Stasinopoulos [44] for parametric GAMLSS models, each model could be assessed by its fitted global deviance (GD) given by

(32) $$\begin{array}{c} \text{GD}=-2l\left(\overset{\wedge }{\theta }\right), \end{array}$$

where $l\left(\overset{\wedge }{\theta }\right)=\sum_{i=1}^{n}l\left(\theta_{i}\right)$.

#### 3.5.3. Bias and Accuracy

The bias measures the average deviation of the predicted value $\overset{\wedge }{f}\left(x\right)$ from the true value *f*(*x*) in a large number of the repeated sampling processes. The bias is often defined as followed given *X*:

(33) $$\begin{array}{c} \text{Bias}\left[\overset{\wedge }{f}\left(x\right)\right]=E\left[\overset{\wedge }{f}\left(x\right)\right]-f\left(x\right). \end{array}$$

MSE can be thought of as measuring the bias of predictions and be defined as

(34) $$\begin{array}{c} \text{MSE}\left[\overset{\wedge }{f}\left(x\right)\right]=E{\left[y-\overset{\wedge }{f}\left(x\right)\right]}^{2}. \end{array}$$

We can prove the MSE is minimized when $\overset{\wedge }{f}\left(x\right)=E\left[y|x\right]$. MSE is obtained through the sample value $\text{MSE}=1/N\sum_{i=1}^{N}{\left({\overset{\wedge }{y}}_{i}-y_{i}\right)}^{2}$, where $\overset{\wedge }{y}$ denotes the estimated and*y* is the true value and *N* is the sample size. The MSE is an unbiased estimator of deviation.

RETRACTED

#### 3.5.4. Out-of-Sample Analysis

There is the last step to examine the appropriateness of the estimated models and the generalization ability of the model. We applied the bootstrap procedure to investigate how the results of our statistical analysis would be generalized to another data set. Given a data set *D* containing *m* samples, we could sample it and generate another data set *D*′. A sample was randomly selected from the data set *D* and put into the data set *D*′, and then the sample was put back into the initial data set *D*, so that the sample might be still drawn next time. After repeating this process *m* times, we were able to get a data set *D*′ consisting of *m* samples. It was obvious that some samples in the data set *D* would appear multiple times in *D*′, while other samples maybe would not appear. The probability that a sample was never selected in *m* sampling was (1 − 1/*m*)^*m*^, and its limit was lim_*m*⟶*∞*_(1 − (1/*m*))^*m*^=1/*e* ≈ 0.368. About 36.8% of the samples in the data set *D* by the bootstrap sampling method did not appear in the sampling data set *D*′. In this way, we could use *D*′ as the training set and (*D* − *D*′) as the test set. In practical application, 1/3 of the sample size was generally selected as test set and 2/3 as the training set.

## 4. Empirical Analysis

### 4.1. Data Description

The aim of this paper was to discover the factors affecting the medical expenditures of the elderly in China and predict the amount using data from the Chinese Longitudinal Healthy Longevity Survey (CLHLS). This survey is a nationally representative panel study, containing observations on individuals aged 65 years or older covering more than half of the counties and cities from 23 provinces, cities, and autonomous regions in China. Since the start of the survey in 1998, it was repeated to follow the same group of the elderly every two or three years, which have been conducted eight waves until 2018. The survey includes questions about the health status, quality of life, medical care, and security needs of the elderly. We used data from the latest survey in 2018, which was a mixed cross-sectional data set collected from 1998 to 2018. In total, the sample consists of 15874 individuals. We finally selected 6832 samples after deleting the data with missing and no response. In what follows, we described variables retained for analysis. We began with the aimed response variable, the medical expenditures, followed by other main independent variables such as income, health, and education.

RETRACTED

### 4.2. Description of Variables

The distribution of medical expenditure for the elderly with the entire sample is shown in Figure 1. We could find that there were a large of zeros, and the histogram of the medical cost was right-skewed and heavily fat tail. From the empirical cumulative distribution plot (Figure 2), it could be seen that the medical expenditure data in the upper right part seriously deviates from the straight line. Therefore, the OLS regression model was not suitable for the data, and other transformed models must be considered. The histogram is shown in Figure 1 suggested a mixture of point distribution and a continuous distribution on the positive side. Consequently, a Tobit model may lead to biased inferences due to there being far more zero observations than expected under the Tobit formulation. The zero-adjusted models offer us a viable framework to deal adequately with the excess of zeros.

For this study, we were interested in revealing the factors affecting medical consumption behavior. In addition to the response variable, we included a set of explanatories in the regressions that turned out to affect the medical expenditure. Typical variables that emerged from the existing literature are age, sex, household income, marriage, and education [1–5]. We incorporated all these variables and added several other variables to the analysis that significantly improved the estimation of the zero-adjusted models. These variables describe the characteristics of the elderly, such as insurance, health status, action limited, individual education, residence, and heart disease or not.

The Andersen Behavioral Model of Health Service Use usually provided a framework for the study of hospitalization that outlined the three determinants: predisposing, enabling, and need factors [48]. In light of this, we evaluated the effects of health status and functional disabilities, as need factors and associated social-demographic factors, as predisposing and enabling factors, on hospitalization utilization. A complete list of the variables used and their descriptive statistics is presented in Table 1. We treated the variables medical expenditure, education, and household income as numerical. For the convenience of calculation, we divided the medical expenditure and the annual household income by 1000. All other variables were categorical and entered into the regressions as dummy variables.

RETRACTED

The density distributions of *f*(*y*), for nonzero medical expenditure are given in Figure 3. In this study, six right-skewed distributions were considered: the normal, student *t*, gamma, inverse Gaussian, generalized gamma and generalized inverse Gaussian distributions. The normal distribution was also presented as a benchmark comparison for the other, right-skewed distributions. All of the candidate distributions were subsequently fitted on a training set of a random 70% subsample. Figure 3 suggested that the normal distribution had the worst fit for the histogram of nonzero medical expenditure and other right-skewed distributions seemed to be fit better. The fitted values of the normal, inverse Gaussian, generalized gamma, and generalized inverse Gaussian distributions underestimated the actual value at the lower points of medical expenditure. However, they showed better fit at other points. The fitted value of the gamma distribution overestimated the lower points. Therefore, there seemed to be no obvious evidence to show which one was the best from the histogram. We must combine other statistical indicators to choose the best model, which was also done in the following section.

## 5. Results

According to the experience above, we chose 4872 samples as training data set.  Table 2 listed the marginal effects estimation results obtained from the training for the models discussed above. We selected ten predictors according to the demand for health and health care of the Grossman model. The estimates of the Tobit model were quite different from others in the value range and sign, which had the largest values of AIC, SBC, and global deviance. This suggested that the Tobit model fitted the data very badly. The new generalized Tobit model and other zero-adjusted models were more similar. Many estimates shared the same sign and had comparable values, resulting in similar conclusions. In terms of the standard errors of the parameters, the errors of the Tobit model were significantly higher than others. All zero-adjusted models had lower standard errors of the parameters. Furthermore, the AIC, SBC, and global deviance (GD) of the zero-adjusted generalized gamma model and zero-adjusted generalized inverse Gaussian model were obviously smaller than those other models. However, the values of the zero-adjusted generalized gamma model were the smallest. The smaller these values are, the better the goodness-fit of the model is. Therefore, the ZAGG model was the best model we chose.

RETRACTED

To assess model fit, we created the quantile residuals plots. If the models were adequate for the data, the residuals approximated a random sample from the standard normal distribution [38].  Figure 4 plots the normalized quantile residuals and shows much difference in the residuals among these models. The residuals of the new generalized Tobit model showed bimodal kurtoses, ZAGA and classic Tobit models presented the aiguille characteristics, and the residuals of the ZAIG model appeared to right-skewed. The residuals of ZAGG and ZAGIG seemed to be similar, but the ZAGG model exhibited a better model fit from Figure 4.

We used worm plots to further study the residuals of these models. Worm plots of the residuals were introduced by van Buuren and Fredriks [49] to identify regions (intervals) of an explanatory variable within which the model does not adequately fit the data. These points in the worm plot, such as Figure 5, showed how far the ordered residuals were from their (approximate) expected values represented by the horizontal dotted line. The closer the points were to the horizontal line, the closer the distribution of the residuals was to a standard normal distribution. Additionally, if the model was correct, we would expect approximately 95% of the points to lie between the two elliptic curves and 5% outside in Figure 5. A higher percentage of the points outside the two elliptic curves indicated that the fitted distribution of the model was inadequate to explain the response variable. The shape of the fitted curve to the points of the worm reflected different inadequacies in the model. A linear trend (positive or negative), quadratic shape (U or inverse U), or cubic shape (S shape) indicated a problem with the variance, skewness, or kurtosis of the residuals, respectively. This, in turn, highlighted a problem with the fitted distribution. Figure 5 shows that the fitted curves of the worm for all models except the zero-adjusted generalized gamma model was S-shaped, which also suggested that the ZAGA model was generally a better fit again.

After the verification of 1960 samples in the test data set, two Tobit models and the ZAIG model had larger MSE values. ZAGG and ZAGIG models again produced very similar results. ZAGIG had the lowest MSE with a value of 671.3679. However, ZAGG was slightly higher with a value of 675.1498 than ZAGIG. Considering the goodness of fit, we chose the ZAGG model for further study.

We chose ZAGG models with different parameters *π*, *σ*, and *ν* and used the default log link function to discover which factors affecting the medical expenditure for the elderly.  Table 3 shows the results of different parameters using 6832 data of the whole population. The predictors for the logarithm of average medical consumption shared almost the same sign and had similar values in the three models. Age, health, and chronic diseases were the main predictors influencing medical expenditure. With the increase of age, the medical expenditure of the elderly was decreasing. Part of the reason might be that the elderly under 80 years old had a higher risk of serious diseases like cancer than the elderly over 80 years old. After experiencing this age stage, most of higher aged elderly were in good health. The elderly in good health had relatively less medical expenditure. As a chronic disease, heart disease significantly increased the medical expenses of the elderly. Compared with the elderly living in cities, the medical expenditure of the elderly living in urban and rural areas was relatively small, which might be related to the relative lack of medical resources in urban and rural areas of China. The higher the family income is, the more the medical expenditure of the elderly is. The predictor of medical insurance value was negative but not significant, which implied that medical insurance maybe reduced the medical expenditure of the elderly and released their financial burden. However, the effect was not obvious.

RETRACTED

The scenario of the ZAGG(I) model: the proportion of *p* of zero medical expenditure and the scale parameter *s* relating to variance were both constant. Because the logit link function was used by default in the regression model, the proportion of zero medical expenditure *π* was 1/(1+exp(1.2984))=0.2144, which was very close to the proportion 0.2147 of zero cost in the population.

The scenario of the ZAGG (II) model: the occurrence of zero medical expenditure varied and was affected by the predictors. We found that some predictors for the medical decision shared different signs. For example, higher values of family income result in lower odds of zero medical expenditure. Perhaps, the elderly with high-income families are more likely to obtain medical resources, and the utilization of medical services was relatively high. The elderly with action limited were often in poor health, so their medical expenditures were more.

The scenario of the ZAGG (III) model: up to now, we had modelled the only *π* as a function of explanatory variables, but there were occasions in which the assumption of a constant scale parameter was not appropriate according to equation (14). On these occasions, modelling *s* as a function of explanatory variables could solve the problem. We could conclude from Figures 6–8 that almost all points of the worm plot failed inside the 95%-pointwise confidence intervals, indicating that the three models appeared to be adequate. Furthermore, the line shape with the negative slope in Figure 6 showed the variance was too low, and the fitted scale was too high. The s-shape with left bent down suggested the tails of fitted distribution was too light.

RETRACTED

Kolmogorov-Smirnov test is a nonparametric test method that can be used to compare the cumulative empirical distributions of two samples. The *D*_*n*_ (*D*_*n*_=sup_*x*_|*F*_*n*_(*x*) − *F*(*x*)|) statistics is used to compare the maximum value of the difference between the empirical distributions of two samples. If this value is too large, we believe that the two distributions are different. Therefore, we used the two tailed Kolmogorov–Smirnov test to verify the consistency between ZAGG model and empirical distribution. The results are shown in the last row of Table 3. From the results, the *p* values were all greater than 0.05, which meant we could not reject the null hypothesis that there was almost no difference between the ZAGG model and empirical distribution.

## 6. Discussion

This paper explored and empirically validated zero-adjusted models with semiparametric formulation for estimating medical expenditures using CLHLS survey data. In reaction to the limitations of conventional Tobit, zero-adjusted gamma, and zero-adjusted inverse Gaussian models, we generalized the three models to improve the accuracy of prediction and discover the factors affecting the elderly medical decision. The zero-adjusted generalized gamma model outperformed the zero-adjusted generalized Tobit and zero-adjusted generalized Inverse Gaussian model. Thus, the ZAGG mode provided an interesting alternative for modelling health care utilization expenditure data as it included many conventional models such as the zero-adjusted Weibull model, the zero-adjusted lognormal model, and the zero-adjusted gamma model. The ZAGG model included log-additive components for the mean and dispersion of medical expenditure given that expenditure occurs, as well as a logistic additive component for the probability of a zero expenditure. The model components were estimated independently and could be fitted with the same set of covariates. In this paper, we firstly chose ZAGG models with different parameters *π*, *σ*, and *ν* and used the default log link function to discover which factors affecting the medical expenditure for the elderly. There was much literature on the influence of factors on the parameter *π*, but there was almost no work discussing the influence of factors on the parameter *σ* and *ν*. We found that some factors might affect the distribution shape and scale change of ZAGG model and then affected the accuracy of the model. These were also contributions of this paper.

RETRACTED

Our empirical application had focused on the assessment of the predictive accuracy and the predictors affecting medical expenditure. We found that ZAGG and ZAGIG gave similar results. Moreover, ZAGG was appreciated for the fact that the generalization errors of ZAGIG were 671.36, which was less than that of ZAGG from mean square errors. However, the ZAGG model seemed to perform better in the aspects of global deviance, AIC and SBC. Whether one of the two models is superior to the other remains an open question, which needs to be determined according to different problems and situations. ZAGG and ZAGIG models, respectively, extended the ZAGA and ZAIG models, and many conventional zero-adjusted models are special forms of these generalized models. Moreover, both of these generalized models increased the difficulty in parameter estimation. For example, the standard errors of parameters were not reliable when the QR decomposition method was used, which could not solve the Hessian matrix. In this paper, we reported the QR-based standard errors using a likelihood-based confidence interval method introduced by Rigby and Stasinopoulos [44, 50, 51].

Although the ZAGG model is complex in application and calculation, it still has some advantages. One benefit of the ZAGG model is that the three components of the mixture model provide the analyst with a three-way interpretation by estimating the factors affecting the medical decision, the factors predicting the amount of the medical expenses, and the factors influencing the dispersion of the expenditure amount. The scale dispersion estimates can be used to provide more conservative estimates when the parameters were less robust. Another advantage of the ZAGG model is that the regression method does not imply a “black box” approach for interpreting the effects of individual covariates. The interpretation of the marginal effect for the model is relatively explicit.

We surprisingly discovered that basic medical insurance had no significant effect on the medical expenditure of the elderly. The main reason was that the basic medical insurance had covered nearly 95% of the population in China up to now, leading to no obvious difference in the impact of medical insurance [2, 52–54]. The elderly with high-income families spent more on health care, which indicated a relatively unfair phenomenon that the poor subsidized the rich in the utilization of medical services in China. At the same time, the medical expenditure in urban and rural areas was relatively low, which also showed that the distribution of medical resources was not balanced.

RETRACTED

Finally, attention should be paid to the limitations of our study. One limitation of this study was that it did not consider the causal relationship between the predictors and response because we were interested in predicting the amount of medical expenditure and unraveled the significant predictors influencing the expenditure. Possible solutions for this causal relationship were either to study only the impact of truly exogenous independent or to apply instrumental variable techniques. Another limitation was that the zero-adjusted models were seemed to be two-stage models, and there existed a variety of models in the continuous part. In this paper, we compared only a few models. Instead, other types of skewed distributions could be considered for further research. Finally, our study has used the two-stage model to predict the amount of medical expenditure. We treated the two parts as independent. However, there perhaps existed a relationship. There were further opportunities to develop potentially superior models by considering the correlation, such as copula function. Moreover, it should be noted that if the relationship were considered, the difficulty of parameter estimation would increase, and the effects of individual explanatory variables could not be interpreted conveniently.

## 7. Conclusions

In this paper, we have predicted the amount of medical expenses for the elderly and explored the marginal effect of the predictors in China, using CLHLS survey data. In reaction to the limitations of conventional Tobit and zero-adjusted models, we generalized these models. This allowed us to estimate the medical expenditure using more flexible models. The zero-adjusted generalized gamma model was the best to fit this data. We focused on the zero-adjusted generalized gamma regression model to reveal the significant factors influencing the medical amount. Several conclusions could be drawn from this work. The health status, family income, residence, and chronic diseases of the elderly significantly affect their medical expenditure, while the influence of basic medical insurance is not significant. We used a logistic model to discover the factors that affected the medical decision of the elderly. We found that the elderly in the higher age group had the lower occurrence of zero medical amount, which indicated they were better health. In addition, this paper accurately estimated the proportion of the elderly with zero medical expenditure using a logit model. In the ZAGG model, we found that the scale dispersion was also affected by the explanatory variables, which could improve the robustness of the standard errors of parameters.

RETRACTED

To the best of our knowledge, this is the first time that using the zero-adjusted generalized gamma model predicts the medical expenditure. The current approach appeared to be effective. However, some limitations merit attention, such as the causal relationship between the predictors and response and the correlations of the two parts in the zero-adjusted models. These limitations required further investigation in the near future.

## Figures and Tables

**Figure 1:** Histogram of medical expenditure.

**Figure 2:** Cumulative distribution of medical expenditure.

**Figure 3:** Candidate distributions for nonzero medical expenditure on the training set. (a) Normal distribution. (b) *t* distribution. (c) Gamma distribution. (d) Inverse Gaussian distribution. (e) Generalized gamma distribution. (f) Generalized inverse Gaussian distribution.

**Figure 4:** Quantile residual for regression models. (a) ZAGA quantile residual. (b) ZAIG quantile residual. (c) ZAGG quantile residual. (d) ZAGIG quantile residual. (e) Generalized Tobit quantile residual. (f) Tobit quantile residual.

**Figure 5:** Worm plots for regression models. (a) ZAGA worm plot. (b) ZAIG worm plot. (c) ZAGG worm plot. (d) ZAGIG worm plot. (e) Generalized Tobit worm plot. (f) Tobit worm plot.

**Figure 6:** Worm plots for ZAGG(I).

**Figure 7:** Worm plots for ZAGG(II).

**Figure 8:** Worm plots for ZAGG(III).

**Table 1:** Descriptive statistics of the dependent and independent variables.

Variable	Description	Mean	S.D	Min	Max
Medical expenditure (numerical)	Medical expenditure/1000	9.034644	25.78056	0	199.998
Gender (categorical)	0 if female	0.4428697	0.4967617	0	1
	1 if male				
Age (categorical)	Age is divided four groups from low to high: lowest = 0 (reference); lower = 1; higher = 2; highest = 3	2.314582	1.129733	1	4
Health (categorical)	Very bad = 0(reference); bad = 1; so so = 2; good = 3; very good = 4	2.449445	0.9057199	0	4
Education (numerical)	Continuous	3.686622	4.413021	0	22
Actlim (categorical)	1 if limited in activities at least the last 6 months	0.3261251	0.4688279	0	1
	0 if not limited (reference)				
Married (categorical)	1 if married	0.4584309	0.4983055	0	1
	0 if divorced, widowed, or never married (reference)				
Insurance (categorical)	1 if participate in any insurance program	0.9211066	0.2695921	0	1
	0 if no insurance (reference)				
Residence (categorical)	1 if current interviewee lived in city (reference)	2.17418	0.8024561	1	3
	2 if lived in town				
	3 if lived in rural				
Heart_disease (categorical)	1 if suffering heart disease	0.1891101	0.3916247	0	1
	0 if no heart disease (reference)				
Household income (numerical)	Household income/1000	42.2063	36.4047	0	99

Note: medical expenses and annual household income are in thousands of yuan.

RETRACTED

**Table 2:** Comparison of marginal effects of Tobit, generated Tobit, ZAGA, ZAIG, ZAGG, and ZAGIG models on CLHLS data.

	Tobit	Generalized Tobit	Zero-adjusted models				
			Discrete	Continuous			
			Binomial	Gamma	Inverse Gaussian	Generalized gamma	Generalized inverse Gaussian
Intercept	17.30660 (4.62914)^∗∗∗^	1.2211352 (0.3509476)^∗∗∗^	−1.214247 (0.441916)^∗∗∗^	3.4395522 (0.2634442)^∗∗∗^	3.131784 (0.980320)^∗∗∗^	1.3507565 (0.3023424)^∗∗∗^	3.3181353 (0.2775036)^∗∗∗^
Gender	−0.12960 (0.93239)	−0.1742161 (0.0706867)^∗∗^	0.107757 (0.081745)	0.1653616 (0.0546928)^∗∗∗^	0.423748 (0.149248)^∗∗∗^	0.0757141 (0.0627683)	0.0798758 (0.0576116)
Age *(lower)*	0.37558 (1.17482)	0.0191777 (0.0890663)	−0.022572 (0.105939)	0.0503636 (0.0683660)	0.094369 (0.184435)	0.0347497 (0.0784604)	0.0439357 (0.0720145)
Age *(higher)*	−2.47297 (1.31612)^*∗*^	−0.1307531 (0.0997782)	0.118543 (0.30750)	−0.0940778 (0.0771663)	−0.063349 (0.200707)	−0.1409848 (0.0885601)	−0.1377442 (0.0812844)^*∗*^
Age *(highest)*	−7.43904 (1.48503)^∗∗∗^	−0.4449018 (0.1125843)^∗∗∗^	0.597306 (0.126676)^∗∗∗^	−0.2929559 (0.0894135)^∗∗∗^	−0.079564 (0.225999)	−0.4639923 (0.1026156)^∗∗∗^	−0.3536105 (0.0941853)^∗∗∗^
Health *(bad)*	−4.90168 (4.18061)	0.4308578 (0.3169431)	−0.466233 (0.413161)	−0.6101187 (0.2364191)^∗∗∗^	−0.331020 (0.924567)	0.0096557 (0.2713270)	−0.3921744 (0.2490362)
Health *(so so)*	−7.88404 (4.09467)^*∗*^	−0.1249660 (0.3104278)	−0.022842 (0.398988)	−0.7872073 (0.2319896)^∗∗∗^	−0.678053 (0.907075)	−0.2875638 (0.2662435)	−0.6390054 (0.2443703)^∗∗∗^
Health *(good)*	−11.95574 (4.11483)^∗∗∗^	−0.4750543 (0.3119565)	0.263264 (0.399472)	−1.1046718 (0.2333300)^∗∗∗^	−1.102426 (0.907025)	−0.7290380 (0.2677818)^∗∗∗^	−0.9737652 (0.2457822)^∗∗∗^
Health *(very good)*	−12.66309 (4.23632)^∗∗∗^	−0.5853829 (0.3211667)^*∗*^	0.291206 (0.407768)	−1.1434518 (0.2410609)^∗∗∗^	−1.076392 (0.918506)	−0.8854640 (0.2766542)^∗∗∗^	−1.1132889 (0.2539257)^∗∗∗^
Education	0.12139 (0.12539)	0.0271759 (0.0095062)^∗∗∗^	−0.016711 (0.011463)	−0.0053850 (0.0073003)	−0.007183 (0.021939)	0.0125635 (0.0083782)	−0.0071493 (0.0076899)
Actlim *(limited)*	6.86144 (0.97959)^∗∗∗^	0.4495150 (0.0742651)^∗∗∗^	−0.589516 (0.091230)^∗∗∗^	0.2587853 (0.0565752)^∗∗∗^	0.200809 (0.152316)	0.4854051 (0.0649287)^∗∗∗^	0.2894195 (0.0595945)^∗∗∗^
Household income	0.09582 (0.01294)^∗∗∗^	0.0025677 (0.0009808)^∗∗∗^	−0.002396 (0.001128)^∗∗∗^	0.0081379 (0.0007603)^∗∗∗^	0.010034 (0.002247)^∗∗∗^	0.0043830 (0.0008726)^∗∗∗^	0.0046224 (0.0008009)^∗∗∗^
Marriage *(married)*	−1.64671 (1.04603)	0.1078140 (0.0793026)	0.005226 (0.092940)	−0.0363325 (0.0612575)	−0.008065 (0.160483)	0.0523691 (0.0703023)	0.0407834 (0.0645266)
Insurance *(insured)*	−5.71764 (1.53651)^∗∗∗^	0.0433423 (0.1164868)	0.020459 (0.133651)	−0.4417009 (0.0904223)^∗∗∗^	−0.296035 (0.260748)	−0.0773757 (0.1037734)	−0.2467232 (0.0952479)^∗∗∗^
Residence *(in town)*	−6.38221 (1.26549)^∗∗∗^	−0.4866704 (0.0959404)^∗∗∗^	0.218619 (0.112552)^*∗*^	−0.5132267 (0.0738881)^∗∗∗^	−0.657867 (0.240905)^∗∗∗^	−0.6409893 (0.0847979)^∗∗∗^	−0.4931939 (0.0778313)^∗∗∗^
Residence *(in rural)*	−5.01228 (1.25786)^∗∗∗^	−0.5029975 (0.0953621)^∗∗∗^	0.055642 (0.112483)	−0.5036751 (0.0733478)^∗∗∗^	−0.693208 (0.238238)^∗∗∗^	−0.8074203 (0.0841778)^∗∗∗^	−0.5935885 (0.0772622)^∗∗∗^
Heart_disease *(suffered)*	8.74595 (1.10292)^∗∗∗^	0.9761225 (0.0836154)^∗∗∗^	−1.139552 (0.132085)^∗∗∗^	0.3834217 (0.0607861)^∗∗∗^	0.503166 (0.198495)^∗∗^	0.6753993 (0.0697614)^∗∗∗^	0.4836672 (0.0640301)^∗∗∗^
*Sigma (σ)*	3.35531 (0.01023)^∗∗∗^	0.37450 (0.02461)^∗∗∗^	—	0.398879 (0.009455)^∗∗∗^	0.30921 (0.01156)^∗∗∗^	0.53659 (0.01156)^∗∗∗^	1.159849 (0.009905)^∗∗∗^
*AIC*	37194.46	27567.15	—	26887.54	26951.03	25575.17	25817.39
*SBC*	37310.97	27690.13	—	27114.08	27177.57	25808.19	26050.41
*GD*	37158.46	27529.15	—	26817.54	26881.03	25503.17	25745.39
*MSE*	702.5649	751.1767	—	675.1498	744.6665	675.1498	671.3679

Note: ( ) indicates the standard errors of the parameters and the stars show the significance of the parameters: ^∗∗∗^*p* < 0.01; ^∗∗^*p* < 0.05; ^*∗*^*p* < 0.1.

RETRACTED

**Table 3:** Results from ZAGG models with different parameters *π*, *σ*, and *ν*.

	ZAGG(I)				ZAGG(II)				ZAGG(III)			
	(*π* and *σ* for constant)				(*π* for all covariates; *σ* for constant)				(*π* and *σ* for all covariates)			
	log(*μ*)	logit(*π*)	log(*σ*)	*ν*	log(*μ*)	logit(*π*)	log(*σ*)	*ν*	log(*μ*)	logit(*π*)	log(*σ*)	*ν*
		−1.2984 (0.0295)^∗∗∗^	0.5412 (0.0097)^∗∗∗^	−0.0215 (0.0196)			0.5412 (0.0097)^∗∗∗^	−0.0215 (0.0196)				−0.0105 (0.0200)
Intercept	1.3922 (0.2488)				1.3922 (0.2489)^∗∗∗^	−1.7032 (0.3400)^∗∗∗^			1.4065 (0.2409)^∗∗∗^	−1.7032 (0.4000)^∗∗∗^	0.4603 (0.1021)^∗∗∗^	
Gender	0.0928 (0.0528)				0.0929 (0.0628)	0.1177 (0.0686)^*∗*^			0.0856 (0.0526)	0.1177 (0.0686)	0.0397 (0.0221)	
Age *(lower)*	0.1085 (0.0656)				0.0347 (0.0785)	−0.0549 (0.0896)			0.0876 (0.0646)	−0.0549 (0.089)	0.0496 (0.0269)^*∗*^	
Age *(higher)*	−0.0960 (0.0740)				−0.1409 (0.0886)	0.1644 (0.0971)^*∗*^			−0.1086 (0.0726)	0.1644 (0.0971)^*∗*^	0.0238 (0.0302)	
Age *(highest)*	−0.3056 (0.0857)^∗∗∗^				−0.4640 (0.1026)^∗∗∗^	0.5715 (0.1068)^∗∗∗^			−0.3019 (0.0867)	0.5715 (0.1068)	0.0571 (0.0345)^*∗*^	
Health *(bad)*	−0.1828 (0.2206)				−0.0957 (0.2713)	0.0097 (0.3771)			−0.2121 (0.2107)	−0.0957 (0.3771)	−0.0001 (0.0911)	
Health *(so so)*	−0.5136 (0.2161)^∗∗^				−0.2876 (0.2662)	0.3518 (0.3658)			−0.5431 (0.2067)^∗∗∗^	0.3517 (0.3658)	0.0182 (0.0891)	
Health *(good)*	−0.9516 (0.2174)^∗∗∗^				−0.7290 (0.2678)^∗∗∗^	0.6387 (0.3660)^*∗*^			−0.9822 (0.2083)^∗∗∗^	0.6387 (0.3660)^*∗*^	0.0412 (0.0894)	
Health *(very good)*	−1.0126 (0.2249)^∗∗∗^				−0.8855 (0.2767)^∗∗∗^	0.7286 (0.3720)^*∗*^			−1.0339 (0.2169)^∗∗∗^	0.7286 (0.3720)^*∗*^	0.0688 (0.0926)	
Education	0.0183 (0.0070)^∗∗∗^				0.0126 (0.0084)	−0.0096 (0.0096)			0.0199 (0.0070)^∗∗∗^	−0.0095 (0.0096)	−0.0024 (0.0029)	
Actlim	0.4699 (0.0540)^∗∗∗^				0.4854 (0.0649)^∗∗∗^	−0.5312 (0.0755)^∗∗∗^			0.47731 (0.0536)^∗∗∗^	−0.5312 (0.0755)^∗∗∗^	−0.00853 (0.0222)	
House hold income	0.0048 (0.0007)^∗∗∗^				0.0044 (0.0009)^∗∗∗^	−0.0031 (0.0010)^∗∗∗^			0.0051 (0.0008)^∗∗∗^	−0.0031 (0.001)^∗∗∗^	0.0014 (0.0003)^∗∗∗^	
Marriage *(married)*	0.0393 (0.0590)				0.0524 (0.0703)	−0.0318 (0.0785)			0.0412 (0.0583)	−0.0318 (0.0785)	−0.0494 (0.0238)^∗∗^	
Insurance *(insured)*	−0.0746 (0.0867)				−0.0774 (0.1038)	0.1055 (0.1145)			−0.0646 (0.0876)	0.1055 (0.1145)	−0.0278 (0.0359)	
Residence *(in town)*	−0.5439 (0.0712)^∗∗∗^				−0.6410 (0.0848)^∗∗∗^	0.2107 (0.0947)^∗∗^			−0.5264 (0.0711)^∗∗∗^	0.2107 (0.0947)^∗∗^	−0.0178 (0.0299)	
Residence *(in rural)*	−0.6579 (0.0702)^∗∗∗^				−0.8074 (0.0842)^∗∗∗^	0.0926 (0.0941)			−0.6408 (0.0712)^∗∗∗^	0.0926 (0.0941)	0.0418 (0.0291)	
Heart_disease *(suffered)*	0.6637 (0.0588)^∗∗∗^				0.6754 (0.0698)^∗∗∗^	−1.1524 (0.1123)^∗∗∗^			0.65708 (0.0569)^∗∗∗^	−1.1524 (0.1123)^∗∗∗^	−0.0459 (0.0242)^*∗*^	
*AIC*	—	37235.64				36845.32				36819.29		
*SBC*	—	37372.23				37091.18				37174.42		
*Dev*	—	37195.64				36773.32				36715.29		
*K-S (D)*		0.012776				0.012171				0.010868		
(*pvalue)*		(0.2147)				(0.2636)				(0.3951)		

Note: () indicates the standard errors of the parameters, and the stars show the significance of the parameters: ^∗∗∗^*p* < 0.01; ^∗∗^*p* < 0.05; ^*∗*^*p* < 0.1.

RETRACTED

## Data Availability

The data in this paper are obtained from the Chinese Longitudinal Healthy Longevity Survey (CLHLS) in 2018.
